# Curcumin Improves Keratinocyte Proliferation, Inflammation, and Oxidative Stress through Mediating the SPAG5/FOXM1 Axis in an *In Vitro* Model of Actinic Dermatitis by Ultraviolet

**DOI:** 10.1155/2022/5085183

**Published:** 2022-09-09

**Authors:** Quan Chen, Yi Tang, Huiyan Deng, Bihua Liang, Huaping Li, Zhenjie Li, Huilan Zhu, Lezi Chen

**Affiliations:** ^1^Guangzhou Institute of Dermatology, Institute of Dermatology, Guangzhou Medical University, No. 56 Hengfu Road, 510095 Guangzhou, Guangdong, China; ^2^Department of Vascular and Plastic Surgery, Guangdong Provincial People's Hospital, Guangdong Academy of Medical Sciences, No. 106 Zhongshan Second Road, 510080 Guangzhou, Guangdong, China

## Abstract

**Background:**

Chronic actinic dermatitis (CAD) is an abnormally proliferating photoallergic skin disease. Dysregulated inflammation and oxidative stress are the immediate factors in the abnormal proliferation of keratinocytes. This study aimed to investigate the effect of curcumin on the aberrant proliferation of keratinocytes in an *in vitro* (actinic dermatitis) AD model and the possible molecular mechanisms.

**Methods:**

The keratinocytes were irradiated with ultraviolet (UV) to construct an *in vitro* AD model and then processed with different concentrations of curcumin. Cell viability, oxidative stress markers (SOD, GSH-PX, and MDA), activated oxygen species (ROS), and inflammation markers (IL-1*β*, IL-6, IL-18, and TNF*α*) were determined, respectively. Western blot was applied to assay the profiles of apoptosis-related proteins (Bax, Bcl-xL, Caspase3, Caspase8, and Caspase9), oxidative stress proteins (Keap1, Nrf2, HO-1, COX2, and iNOS), and inflammatory proteins (NF-*κ*B, MMP1, and MMP9) and SPAG5/FOXM1. Functionally, SPAG5 or FOXM1 overexpression and knockdown models were constructed in keratinocytes to characterize their influence on UV irradiation-mediated keratinocyte dysfunction.

**Results:**

Curcumin weakened UV-mediated inflammation, proliferation, and oxidative stress and impaired apoptosis in keratinocytes. UV boosted SPAG5/FOXM1 expression in cells, while curcumin concentration-dependently retarded SPAG5/FOXM1 expression. Overexpression of SPAG5/FOXM1 fostered UV-mediated inflammation, proliferation, oxidative stress, and intensified apoptosis, whereas curcumin mostly reversed the SPAG5/FOXM1-mediated effects. In addition, knocking down SPAG5/FOXM1 ameliorated UV-mediated keratinocyte dysfunction, whereas curcumin failed to exert further protective effects in cells with knockdown of SPAG5/FOXM1.

**Conclusion:**

Curcumin modulated proliferation, inflammation, oxidative stress, and apoptosis of keratinocytes by restraining the SPAG5/FOXM1 axis.

## 1. Introduction

Chronic actinic dermatitis (CAD) is a photoallergic disorder caused by ultraviolet A (UVA), ultraviolet B (UVB), or visible light [1]. CAD is most often seen in middle-aged and older men who have been exposed to the sun for many years and is typically characterized by pruritic eczema and mossy plaques with markedly reduced skin folds in sun-exposed areas, including the chin, the area behind the ears, and the nasolabial folds [2]. The treatment of CAD requires avoidance of light and exposure to well-defined allergenic substances and medications, strict sun protection when going out, and sometimes the necessity to avoid outdoor activities altogether, which seriously affects the patients' quality of life [3, 4]. There is no curative treatment for CAD currently [5]; it is imperative to develop novel strategies for CAD treatment.

Curcumin is the predominant active ingredient in *Curcuma longa* with pronounced anti-inflammatory, antioxidant, antitumor, anticoagulant, and anti-infective effects [6]. As reported, curcumin mitigates oxidative stress and apoptosis in UVB-irradiated HaCaT cells by diminishing reactive oxygen species (ROS) levels and curbing the mitochondrial pathway [7]. Curcumin exhibits anti-inflammatory effects in acute skin inflammation by restraining COX-2 expression in UVB-irradiated human keratinocytes (HaCaT) through blocking the activity of p38 MAPK and JNK [8]. In parallel, curcumin restricts UVB-induced growth and proliferation of keratinocytes by enhancing p53 phosphorylation through the activation of p38 MAP kinase [9]. Nonetheless, the molecular mechanisms by which curcumin alleviates ultraviolet- (UV-) mediated keratinocyte dysfunction await further investigation.

Sperm-associated antigen 5 (SPAG5) is a mitotic spindle protein that is implicated in cell proliferation, apoptosis, and autophagy [10]. Increased SPAG5 expression is linked to unfavorable prognosis in glioma patients. Knockout of SPAG5 restrains proliferation, colony formation, migration, and invasion of glioma cells and stimulates apoptosis [11]. Forkhead box M1 (FOXM1) belongs to the Forkhead family, which is a transcription factor associated with cell proliferation [12]. Low-power laser irradiation (LPLI) delays UVB-induced cellular senescence by activating extracellular regulated protein kinases (ERKs) to facilitate the phosphorylation of FOXM1 and nuclear translocation to downregulate p21 [13]. Previous studies have revealed that SPAG5 silencing decreases matrix metalloproteinase-2 (MMP2) expression by downregulating FOXM1 to curb osteosarcoma (OS) cell invasion, migration, metastasis, and epithelial-mesenchymal transition (EMT) [14]. Nevertheless, the mechanism of action of SPAG5/FOXM1 in CAD is elusive.

In the present study, HaCaT cells were subject to UV irradiation to develop an *in vitro* actinic dermatitis (AD) model and discovered that curcumin abated the proliferation, inflammation, oxidative stress, and apoptosis of UV-irradiated keratinocytes and hindered the SPAG5/FOXM1 pathway. Overexpression of SPAG5/FOXM1 worsened UV irradiation-mediated keratinocyte dysfunction, which was ameliorated by knockdown of SPAG5/FOXM1. In conclusion, curcumin exerts keratinocyte-protective effects via repression of the SPAG5/FOXM1 pathway in an *in vitro* AD model.

## 2. Materials and Methods

### 2.1. Cell Culture

HaCaT cells were obtained from American Type Culture Collection (Manassas, VA, USA). Cells were cultured in Dulbecco's Modified Eagle's Medium (Invitrogen, Carlsbad, CA, USA) comprising 10% fetal bovine serum (Invitrogen), 100 U/mL penicillin (Invitrogen), and 100 U/mL streptomycin (Sigma-Aldrich, St. Louis, MO, USA) and maintained in a humidified incubator at 37°C with 5% CO_2_.

### 2.2. Cell Transfection

The HaCaT cells were plated into a 6-well plate. Next day, SPAG5 overexpression plasmid, FOXM1 overexpression plasmid, control vector, si-SPAG5, si-FOXM1, and si-NC were transfected into HaCaT cells individually using Lipofectamine 3000 (Invitrogen, USA) according to the manufacturer's instructions.

### 2.3. UV Irradiation and Drug Treatment

The medium was substituted with phosphate-buffered saline (PBS, 200 *μ*L/well), and HaCaT cells were then exposed to UVB radiation (range: 280–315 nm; dose: 50 mJ/cm^2^; duration: 45 min) with the aid of a BIO-LINK crosslinker (BLX; Vilber Lourmat, Collégien, France). Following UVB irradiation, the cells were flushed with PBS and cultured for 24 hours in a fresh medium. UVB-induced HaCaT cells were then processed with curcumin (2.5, 5 *μ*M) for 24 hours.

### 2.4. The Cell Counting Kit-8 (CCK-8) Assay

The CCK-8 experiment was used to determine cell viability. HaCaT cells from each treatment group were inoculated in 96-well plates at 1 × 10^3^ cells per well. After 24 hours of incubation, 10 *μ*L CCK-8 solution was added to each well and kept at 37°C with 5% CO_2_ for 2 hours. The absorbance at 450 nm was monitored using a Multiskan Spectrum (Thermo Fisher Scientific, USA).

### 2.5. Reverse Transcriptase-Polymerase Chain Reaction (RT-PCR)

Total RNA was extracted from HaCaT cells using the RNeasy Mini Kit (Qiagen, Hilden, Germany) following the manufacturer's instructions. The cDNA was synthesized by utilizing the iScript cDNA synthesis kit (Bio-Rad, Hercules, CA, USA). Taq Pro Universal SYBR qPCR Master Mix (Vazyme, Jiangsu, China) was applied in a Step-One Plus Real-Time PCR System (Foster City, CA, USA) to determine the expression of SPAG5, FOXM1, IL-1*β*, IL-6, IL-18, and TNF*α*. The program was 95°C for 30 s, 40 cycles of 95°C for 10 s, and 60°C for 30 s. Calculations were carried out using the 2^−∆∆CT^ method. The primer sequences are listed in Table 1.

### 2.6. Western Blot

Proteins in cells were isolated with the NEPER Nuclear and Cytoplasmic Extraction Kit (Thermo Fisher Scientific, Waltham, MA, USA). Protein concentrations were measured using the BCA Protein Assay Kit (Thermo Fisher Scientific). Total protein (30 *μ*g) was separated on sodium dodecyl sulfate, sodium salt-polyacrylamide gel electrophoresis (SDS-PAGE) and transferred to polyvinylidene fluoride (PVDF) membranes (Millipore, Bedford, MA, USA). The membranes were blocked with 5% skim milk for 2 hours and incubated with primary antibodies such as anti-Bax (Abcam, 1 : 1000, ab32503, Shanghai, China), anti-Bcl-xL (Abcam, 1 : 1000, ab32370), anti-C-Caspase3 (Abcam, 1 : 1000, ab32042), anti-C-Caspase8 (Thermo Fisher Scientific, 1 : 1000, MA5-38680, Massachusetts, USA), anti-C-Caspase9 (Abcam, 1 : 1000, ab2324), anti-Keap1 (Abcam, 1 : 1000, ab139729) (Abcam, 1 : 1000, ab62352), anti-Nrf2 (Abcam, 1 : 1000, ab62352), anti-HO-1 (Abcam, 1 : 1000, ab52947), anti-COX2 (Abcam, 1 : 1000, ab62331), anti-iNOS (Abcam, 1 : 1000, ab178945), anti-p-NF-*κ*B (Abcam, 1: 1000, ab76302), anti-NF-*κ*B (Abcam, 1 : 1000, ab32360), anti-MMP1 (Abcam, 1 : 1000, ab134184), anti-MMP9 (Abcam, 1 : 1000, ab228402), anti-SPAG5 (Abcam, 1 : 1000, ab241581), anti-FOXM1 (Abcam, 1 : 1000, ab207298), and anti-GAPDH (Abcam, 1 : 1000, ab9485) overnight at 4°C. Subsequently, the membranes were incubated with horseradish peroxidase-labeled secondary antibodies for 2 hours at 37°C. Finally, protein-antibody complexes were identified with the ECL detection kit (Millipore). The ImageJ software (National Institutes of Health, Bethesda, MD, USA) was employed for protein quantification.

### 2.7. Reactive Oxygen Species (ROS) Detection

HaCaT cells were inoculated in 24-well plates for 24 hours and then subjected to incubation with 10 *μ*M 2′,7′-dichlorodihydrofluorescein diacetate (DCFH-DA) in a serum-free DMEM for 20 minutes away from light. After incubation, the cells were cleared with serum-free DMEM and the fluorescence intensity was checked with a fluorescent microscope (Leica, Germany). Finally, the ROS level was determined with the fluorescence level.

### 2.8. The Detection of SOD, GSH-PX, and MDA Levels

HaCaT cells were inoculated in 6-well plates at 1.5 × 10^5^/per well and incubated overnight. Then, the cells were collected from each treatment group, flushed, and lysed in liquid nitrogen. The levels of SOD, GSH-PX, and MDA in the cells were estimated using the Oxidative Stress Assay Kit (Beyotime, Shanghai, China) based on the manufacturer's description.

### 2.9. Statistics and Analysis

Experimental results were presented as mean ± SD. Data analysis was performed using the SPSS 22.0 software (IBM, Armonk, NY, USA). The measures were analyzed by ANOVA, and statistical significance was determined by *t*-test or ANOVA. The two-sided *p* < 0.05 was regarded as statistically significant.

## 3. Results

### 3.1. Curcumin Lessened Proliferation, Inflammation, Oxidative Stress, and Apoptosis in UV-Irradiated Keratinocytes

To determine the function of curcumin in AD, we built an *in vitro* AD model using UV-irradiated HaCaT cells and then treated the cells with 2.5 *μ*M and 5 *μ*M of curcumin for 24 hours, respectively. The CCK-8 assay displayed that UV irradiation enhanced HaCaT cell proliferation in comparison to the CON group, while curcumin treatment restrained the proliferative viability of UV-irradiated HaCaT cells (Figure 1(a)). The findings of the Oxidative Stress Assay Kit highlighted that UV-irradiated HaCaT cells had declined contents of SOD and GSH-PX and raised levels of MDA compared to the CON group. Curcumin treatment uplifted the levels of SOD and GSH-PX and decreased the MDA content in UV-irradiated HaCaT cells versus the UV group (Figures 1(b)– 1(d)). Cell fluorescence assays displayed elevated levels of ROS in UV-irradiated HaCaT cells compared to the CON group, while curcumin administration choked the levels of ROS (Figure 1(e)). As testified by RT-PCR outcomes, UV irradiation enhanced the expression of inflammatory factors IL-1*β*, IL-6, IL-18, and TNF*α* in HaCaT cells versus the Con group, and curcumin processing dampened the expression of these inflammatory factors in UV-irradiated HaCaT cells (Figure 1(f)). WB results displayed elevated expressions of Bax, Caspase3, Caspase8, Caspase9, Keap1, COX2, iNOS, NF-*κ*B, MMP1, and MMP9 and diminished expressions of Bcl-xL, Nrf2, and HO-1 in UV-irradiated HaCaT cells compared to the CON group, and curcumin treatment reversed these effects (Figures 1(g)– 1(i)). In addition, we observed that the effect of 5 *μ*M curcumin was obviously stronger than that of 2.5 *μ*M curcumin (Figures 1(a)– 1(i)). Thus, curcumin abated proliferation, inflammation, oxidative stress, and apoptosis in UV-irradiated keratinocytes.

### 3.2. Curcumin Inactivated the SPAG5/FOXM1 Pathway

To measure the expression characteristics of the SPAG5/FOXM1 pathway in an *in vitro* AD model, we assayed the expression of SPAG5 and FOXM1 in UV-irradiated HaCaT cells by WB and RT-PCR. As a result, UV irradiation facilitated the profiles of SPAG5 and FOXM1 in HaCaT cells versus the CON group, and curcumin presented a concentration-dependent inhibition of the SPAG5/FOXM1 pathway expression in UV-irradiated HaCaT cells (Figures 2(a) and 2(b)). Hence, curcumin choked the SPAG5/FOXM1 pathway.

### 3.3. Overexpression of SPAG5 Fostered UV Irradiation-Mediated Keratinocyte Dysfunction

To evaluate into the function of SPAG5 in AD, we transfected vectors and SPAG5 overexpression plasmids into HaCaT cells and assayed the SPAG5 expression in HaCaT cells by RT-PCR 24 hours later. The findings presented that HaCaT cells transfected with the SPAG5 overexpression plasmids had an elevated expression of SPAG5 compared to the vector group (Figure 3(a)). Next, we administered UV irradiation to the transfected HaCaT cells and then manipulated them with curcumin (5 *μ*M) for 24 hours. As verified by CCK-8 results, overexpression of SPAG5 facilitated the proliferative viability of UV-irradiated HaCaT cells. In parallel, the addition of curcumin in the SPAG5 + UV group contributed to the diminished proliferation of HaCaT cells (Figure 3(b)). Oxidative stress assay kits and cytofluorimetric assays displayed that SPAG5 overexpression decreased SOD and GSH-PX levels and uplifted MDA and ROS contents in UV-irradiated HaCaT cells. Meanwhile, the concentrations of SOD and GSH-PX were raised and the levels of MDA and ROS were declined in the SPAG5 + UV + curcumin group compared to the SPAG5 + UV group (Figures 3(c)– 3(f)). RT-PCR results revealed that SPAG5 overexpression boosted the expression of inflammatory factors (IL-1*β*, IL-6, IL-18, TNF*α*) in UV-irradiated HaCaT cells. In contrast, the profiles of inflammatory factors were signally lower in HaCaT cells in the SPAG5 + UV + curcumin group versus the SPAG5 + UV group (Figure 3(g)). WB displayed that overexpressing SPAG5 upregulated Bax, Caspase3, Caspase8, Caspase9, Keap1, COX2, iNOS, NF-*κ*B, MMP1, MMP9, SPAG5, and FOXM1 and downregulated Bcl-xL, Nrf2, and HO-1 in UV-irradiated HaCaT cells, whereas curcumin treatment diminished these effects (Figures 3(h)– 3(k)). In summary, overexpression of SPAG5 potentiated UV irradiation-mediated keratinocyte dysfunction, and curcumin reversed the effects mediated by SPAG5 overexpression.

### 3.4. Overexpressing FOXM1 Accelerated UV Irradiation-Mediated Dysfunction of Keratinocytes

To determine the function of FOXM1 in AD, we transfected vectors and FOXM1 overexpression plasmids into HaCaT cells and assayed the transfection efficiency by RT-PCR after 24 hours. As a result, the expression of FOXM1 was notably augmented in HaCaT cells in the FOXM1 group versus the vector group (Figure 4(a)). Next, we treated transfected HaCaT cells with UV irradiation and then with 5 *μ*M curcumin for 24 hours. As disclosed by CCK-8 outcomes, overexpressing FOXM1 enhanced the proliferative viability of UV-irradiated HaCaT cells versus the UV group. The proliferation of HaCaT cells was restricted in the FOXM1 + UV + curcumin group compared to the FOXM1 + UV group (Figure 4(b)). The results of the oxidative stress assay kit and cytofluorimetry hinted that the levels of SOD and GSH-PX were reduced and the contents of MDA and ROS were uplifted in UV-irradiated HaCaT cells after overexpression of FOXM1. In parallel, as compared to the FOXM1 + UV group, the FOXM1 + UV + curcumin group exhibited elevated levels of SOD and GSH-PX and reduced levels of MDA and ROS in HaCaT cells (Figures 4(c)– 4(f)). RT-PCR results indicated that the levels of inflammatory factors IL-1*β*, IL-6, IL-18, and TNF*α* were heightened in HaCaT cells in the FOXM1 + UV group versus the UV group. The administration of curcumin to the FOXM1 + UV group resulted in a declined expression of inflammatory factors in HaCaT cells (Figure 4(g)). As validated by WB outcomes, overexpressing FOXM1 facilitated the expression of Bax, Caspase3, Caspase8, Caspase9, Keap1, COX2, iNOS, NF-*κ*B, MMP1, MMP9, and FOXM1 and retarded the expression of Bcl-xL, Nrf2, and HO-1 in UV-irradiated HaCaT cells without affecting the expression of SPAG5 significantly, whereas curcumin treatment abated these effects (Figures 4(h)– 4(k)). These results hinted that overexpressing FOXM1 contributed to proliferation, inflammation, oxidative stress, and apoptosis in UV-irradiated keratinocytes, whereas curcumin largely reversed the effects mediated by FOXM1 overexpression.

### 3.5. Knocking Down SPAG5 Ameliorated UV-Irradiated Keratinocyte Dysfunction

To further exploit the role of SPAG5 in AD, we transfected si-NC and si-SPAG5 into HaCaT cells. The SPAG5 expression in transfected HaCaT cells was checked by RT-PCR after 24 hours, which displayed that SPAG5 was remarkably downregulated in HaCaT cells in the si-SPAG5 group versus the si-NC group (Figure 5(a)). We then exposed the transfected HaCaT cells to UV irradiation and treated them with 5 *μ*M curcumin for 24 hours. The CCK-8 assay illustrated that knocking down SPAG5 curbed the proliferative viability of UV-irradiated HaCaT cells. Treatment with curcumin based on the si − SPAG5 + UV group had no remarkable impact on HaCaT cell proliferation (Figure 5(b)). The results of the oxidative stress assay kit and cytofluorimetry disclosed that knockdown of SPAG5 heightened the levels of SOD and GSH-PX and hindered the contents of MDA and ROS in UV-irradiated HaCaT cells compared to the UV group. In parallel, the levels of SOD, GSH-PX, MDA, and ROS were not significantly altered in HaCaT cells in the si − SPAG5 + UV + curcumin group versus the si − SPAG5 + UV + curcumin group (Figures 5(c)– 5(f)). As demonstrated by RT-PCR findings, knockdown of SPAG5 restrained the expression of inflammatory factors IL-1*β*, IL-6, IL-18, and TNF*α* in UV-irradiated HaCaT cells. Meanwhile, curcumin treatment did not influence the expression of inflammatory factors in UV-irradiated HaCaT cells after knockdown of SPAG5 compared to the si − SPAG5 + UV group (Figure 5(g)). Also, WB results confirmed that knockdown of SPAG5 downregulated Bax, Caspase3, Caspase8, Caspase9, Keap1, COX2, iNOS, NF-*κ*B, MMP1, MMP9, SPAG5, and FOXM1 and upregulated Bcl-xL, Nrf2, and HO-1 in UV-irradiated HaCaT cells compared to the UV group. Nevertheless, there was no significant difference in the expression of the above proteins in HaCaT cells in the si − SPAG5 + UV group versus the si − SPAG5 + UV + curcumin group (Figures 5(h)– 5(k)). Thus, knockdown of SPAG5 alleviated UV irradiation-mediated keratinocyte dysfunction.

### 3.6. Knockdown of FOXM1 Eased UV Irradiation-Mediated Dysfunction of Keratinocytes

To further investigate the function of FOXM1 in AD, we transfected si-NC and si-FOXM1 into HaCaT cells. The transfection efficiency was checked by RT-PCR after 24 hours, which highlighted that the expression of FOXM1 was declined in HaCaT cells after transfection with si-FOXM1 compared to the si-NC group (Figure 6(a)). Next, we treated the transfected HaCaT cells with UV irradiation and then with curcumin (5 *μ*M) for 24 hours. As uncovered by CCK-8 results, the proliferation of HaCaT cells was impaired in the si − FOXM1 + UV group versus the UV group. Meanwhile, curcumin treatment did not influence the proliferation of UV-irradiated HaCaT cells after knockdown of FOXM1 versus the si − FOXM1 + UV group (Figure 6(b)). Oxidative stress assay kits and cytofluorimetric assays demonstrated that knockdown of FOXM1 elevated SOD and GSH-PX levels and choked MDA and ROS contents in UV-irradiated HaCaT cells. There was no major disparity in the levels of SOD, GSH-PX, MDA, and ROS between the si − FOXM1 + UV group and the si − FOXM1 + UV + curcumin group of HaCaT cells (Figures 6(c)– 6(f)). RT-PCR uncovered that knockdown of FOXM1 hindered the expression of inflammatory factors (IL-1*β*, IL-6, IL-18, and TNF*α*) in UV-irradiated HaCaT cells. In contrast, the expression of inflammatory factors in HaCaT cells was not distinctly altered in the si − FOXM1 + UV + curcumin group in comparison to the si − FOXM1 + UV + curcumin group (Figure 6(g)). As disclosed by WB results, Bax, Caspase3, Caspase8, Caspase9, Keap1, COX2, iNOS, NF-*κ*B, MMP1, MMP9, and FOXM1 were downregulated and Bcl-xL, Nrf2, and HO-1 were upregulated in the si − FOXM1 + UV group of HaCaT cells compared to the UV group, while the expression of SPAG5 was not significantly altered. Treatment with curcumin on the basis of the si − FOXM1 + UV group restrained the expression of SPAG5 in HaCaT cells, while it had no notable impact on the expression of other proteins (Figure 6(h)– 6(k)). These results demonstrated that knockdown of FOXM1 ameliorated UV irradiation-mediated dysfunction of keratinocytes.

## 4. Discussion

CAD is an immune-mediated photodermatosis. As the disease progresses, the lesioned skin becomes rough and thickened, with mossy lesions and increased pruritus, and patients may even scratch the skin and suffer complications such as local skin infections and artificial dermatitis [15, 16]. Here, we demonstrated that curcumin diminishes proliferation, inflammation, oxidative stress, and apoptosis of keratinocytes via repression of the SPAG5/FOXM1 axis in an *in vitro* AD model.

UV is the light in sunlight with a wavelength of 10 nm to 400 nm and can be classified as UVA, UVB, and UVC. UV is not visible as it lies outside of the violet light in the spectrum [17]. Excessive exposure of the skin to UV radiation causes oxidative stress, inflammation, immunosuppression, matrix metalloproteinase production, and DNA damage and mutations, resulting in skin photodamage [18]. Corneocytes, the main functional and structural component of the epidermis, account for more than 80% of epidermal cells and are the first line of defense against UV radiation [19, 20]. Here, we constructed an *in vitro* AD model in UV-irradiated HaCaT cells and observed that UV irradiation dramatically stimulated oxidative stress and inflammatory responses in HaCaT cells compared to controls.

Curcumin is a natural compound isolated from *Curcuma longa*, which exerts an essential role in inflammatory, neoplastic, and infectious skin diseases [21]. For instance, curcumin protects HaCaT cells from UV irradiation-induced photodamage by activating nuclear factor erythroid 2-related factor 2 (Nrf2) to restrain apoptosis and oxidative stress [22]. Curcumin protects the skin from UVB-induced epidermal cytotoxicity by triggering the Keap1-Nrf2 pathway [23]. Curcumin suppresses oxidative stress in acute UVB-irradiated immortalized human keratinocytes (HaCaT) through activation of Nrf2 and exerts a photoprotective effect in acute photodamage [24]. Our findings are concordant with previous studies where we discovered that curcumin treatment substantially increased the proliferation, inflammation, oxidative stress, and apoptosis of UV-irradiated keratinocytes with higher concentrations of curcumin having a more pronounced effect.

SPAG5 is an emerging oncogene that is overexpressed and exerts carcinogenic effects in diverse cancers such as lung adenocarcinoma [25] and liver cancer [26]. In diabetic nephropathy, lncRNA SPAG5-AS1 activates the AKT/mTOR pathway through upregulation of SPAG5 to foster apoptosis and abate autophagy in high glucose- (HG-) treated human podocytes (HPCs) [27]. FOXM1 is a novel tumor biomarker that is involved in modulating psoriasis [28], keloid [29], and many other skin diseases. FOXM1 is notably upregulated in psoriatic skin tissues and in TNF*α*-stimulated HaCaT cells. FOXM1 knockout curbs TNF*α*-induced proliferation and inflammatory response of HaCaT cells and potentiates apoptosis by restraining the NF-*κ*B pathway [30]. A study has revealed that downregulation of SPAG5 suppresses the ADAM17/NOTCH1 pathway by lowering the expression of FOXM1 in malignant melanoma (MM), thereby dampening the viability, migration, invasion, and EMT of MM cells [31]. Nevertheless, the involvement of the SPAG5/FOXM1 pathway in AD is unclear. In the present research, we identified that UV contributed to the expression of the SPAG5/FOXM1 pathway, while curcumin concentration-dependently restrained the SPAG5/FOXM1 pathway. Overexpression of SPAG5/FOXM1 facilitated UV irradiation-mediated dysfunction in keratinocytes, whereas curcumin mostly reversed the effects mediated by SPAG5/FOXM1 overexpression. Knockdown of SPAG5/FOXM1 ameliorated UV irradiation-mediated keratinocyte dysfunction and counteracted the protective effect of curcumin on keratinocytes.

Overall, our study illustrates that curcumin protects keratinocytes from UV irradiation-induced photodamage by modulating the SPAG5/FOXM1 axis in an *in vitro* AD model. Our findings shed light on new ideas and directions for the treatment of AD.

## Figures and Tables

**Figure 1:** Curcumin reduced proliferation, inflammation, oxidative stress, and apoptosis in UV-irradiated keratinocytes. An *in vitro* AD model was constructed in UV-irradiated HaCaT cells, which were then treated with 2.5 *μ*M and 5 *μ*M curcumin for 24 hours. (a) HaCaT cell proliferation was measured by CCK-8. (b)–(d) The levels of SOD, GSH-PX, and MDA in HaCaT cells were gauged with an oxidative stress assay kit. (e) The ROS content in HaCaT cells was assessed by cytofluorimetry. (f) Expression of inflammatory factors IL-1*β*, IL-6, IL-18, and TNF*α* in HaCaT cells was compared by ELISA. (g) The profiles of apoptosis-related proteins Bax, Bcl-xL, Caspase3, Caspase8, and Caspase9 in HaCaT cells were assayed by WB. (h) WB was conducted to measure the expression of oxidative stress-related proteins Keap1, Nrf2, HO-1, COX2, and iNOS in HaCaT cells. (i) Expression of inflammation-related proteins NF-*κ*B, MMP1, and MMP9 in HaCaT cells was determined by WB. *N* = 3. ∗*p* < 0.05 (vs. CON group), ∗∗*p* < 0.01, ∗∗∗*p* < 0.001; ^#^*p* < 0.05 (vs. UV group), ^##^*p* < 0.01, ^###^*p* < 0.001.

**Figure 2:** Curcumin choked the SPAG5/FOXM1 pathway. (a) Expression of SPAG5 and FOXM1 in HaCaT cells was probed by WB. (b) RT-PCR was implemented to verify the profiles of SPAG5 and FOXM1 mRNA in HaCaT cells. *N* = 3. ∗*p* < 0.05 (vs. CON group), ∗∗*p* < 0.01, ∗∗∗*p* < 0.001; ^#^*p* < 0.05 (vs. UV group), ^##^*p* < 0.01, ^###^*p* < 0.001.

**Figure 3:** Overexpression of SPAG5 potentiated UV irradiation-mediated dysfunction of keratinocytes. (a) Vectors and SPAG5 overexpression plasmids were transfected into HaCaT cells, and the SPAG5 expression in HaCaT cells was assayed by RT-PCR 24 hours later. The transfected HaCaT cells were irradiated with UV and then treated with curcumin (5 *μ*M) for 24 hours. (b) CCK-8 was applied to check the proliferation of UV-irradiated HaCaT cells. (c)–(f) Levels of SOD, GSH-PX, MDA, and ROS in UV-irradiated HaCaT cells were assessed using an oxidative stress assay kit and cytofluorimetry. (g) ELISA tested the expression of inflammatory factors IL-1*β*, IL-6, IL-18, and TNF*α* in UV-irradiated HaCaT cells. (h)–(j) WB was conducted to investigate the profiles of apoptosis-associated proteins (Bax, Bcl-xL, Caspase3, Caspase8, Caspase9), oxidative stress-associated proteins (Keap1, Nrf2, HO-1, COX2, iNOS), and inflammatory response proteins (NF-*κ*B, MMP1, MMP). (k) The expression of the SPAG5/FOXM1 pathway in UV-irradiated HaCaT cells was estimated by WB. *N* = 3. ∗*p* < 0.05 (vs. vector or UV group), ∗∗*p* < 0.01, ∗∗∗*p* < 0.001; ^#^*p* < 0.05 (vs. SPAG5+UV group), ^##^*p* < 0.01, ^###^*p* < 0.001.

**Figure 4:** Overexpression of FOXM1 stimulated UV irradiation-mediated dysfunction of keratinocytes. (a) Vectors and FOXM1 overexpression plasmids were transfected into HaCaT cells, and the transfection efficiency was inspected by RT-PCR after 24 hours. The transfected HaCaT cells were then subjected to UV irradiation and treated with 5 *μ*M curcumin for 24 hours. (b) UV-irradiated HaCaT cell proliferation was assayed using CCK-8. (c)–(e) Levels of SOD, GSH-PX, and MDA in UV-irradiated HaCaT cells were compared using the Oxidative Stress Assay Kit. (f) The amount of ROS in UV-irradiated HaCaT cells was determined by cytofluorimetry. (g) ELISA was implemented to verify the profiles of inflammatory factors (IL-1*β*, IL-6, IL-18, TNF*α*) in UV-irradiated HaCaT cells. (h)–(k) Expression of Bax, Bcl-xL, Caspase3, Caspase8, Caspase9, Keap1, Nrf2, HO-1, COX2, iNOS, NF-*κ*B, MMP1, MMP9, SPAG5, and FOXM1 in UV-irradiated HaCaT cells was examined with WB. *N* = 3. ∗*p* < 0.05 (vs. vector or UV group), ∗∗*p* < 0.01, ∗∗∗*p* < 0.001; ^#^*p* < 0.05 (vs. FOXM1+UV group), ^##^*p* < 0.01, ^###^*p* < 0.001.

**Figure 5:** Knockdown of SPAG5 ameliorated UV irradiation-mediated dysfunction of keratinocytes. (a) The si-NC and si-SPAG5 were transfected into HaCaT cells and the expression of SPAG5 was evaluated by RT-PCR 24 hours later. We then exposed the transfected HaCaT cells to UV irradiation and treated them with 5 *μ*M curcumin for 24 hours. (b) UV-irradiated HaCaT cell proliferation was assayed with CCK-8. (c)–(f) The levels of SOD, GSH-PX, MDA, and ROS in UV-irradiated HaCaT cells were tested using an oxidative stress assay kit and cytofluorimetry. (g) Expression of inflammatory factors (IL-1*β*, IL-6, IL-18, and TNF*α*) in UV-irradiated HaCaT cells was checked by RT-PCR. (h) Expression of apoptosis-related proteins (Bax, Bcl-xL, Caspase3, Caspase8, Caspase9) in UV-irradiated HaCaT cells was detected by WB. (i) WB was implemented to testify the profiles of oxidative stress-related proteins (Keap1, Nrf2, HO-1, COX2, and iNOS) in UV-irradiated HaCaT cells. (j) The expression of inflammatory response proteins (NF-*κ*B, MMP1, and MMP9) in UV-irradiated HaCaT cells was evaluated by WB. (k) The SPAG5/FOXM1 pathway expression in UV-irradiated HaCaT cells was testified by WB. *N* = 3. ∗*p* < 0.05 (vs. si-NC or UV group), ∗∗*p* < 0.01, ∗∗∗*p* < 0.001; ^#^*p* < 0.05 (vs. si-SPAG5+UV group), ^##^*p* < 0.01, ^###^*p* < 0.001.

**Figure 6:** Knockdown of FOXM1 alleviated UV irradiation-mediated dysfunction of keratinocytes. (a) si-NC and si-FOXM1 were transfected into HaCaT cells and transfection efficiency was measured by RT-PCR after 24 hours. The transfected HaCaT cells were processed by UV irradiation and then treated with curcumin (5 *μ*M) for 24 hours. (b) CCK-8 was employed to examine the proliferation of UV-irradiated HaCaT cells. (c)–(e) The contents of SOD, GSH-PX, and MDA in UV-irradiated HaCaT cells were evaluated using the Oxidative Stress Assay Kit. (f) Cytofluorimetry was applied to assay the level of ROS in UV-irradiated HaCaT cells. (g) The expression of inflammatory cytokines in UV-irradiated HaCaT cells was monitored by RT-PCR. (h) WB was adopted to verify the expression of apoptosis-related proteins in UV-irradiated HaCaT cells. (i) WB gauged the expression of oxidative stress-related proteins in UV-irradiated HaCaT cells. (j) The profiles of inflammatory response proteins in UV-irradiated HaCaT cells were compared by WB. (k) WB assessed the SPAG5/FOXM1 pathway expression in UV-irradiated HaCaT cells. *N* = 3. ∗*p* < 0.05 (vs. si-NC or UV group), ∗∗*p* < 0.01, ∗∗∗*p* < 0.001; ^#^*p* < 0.05 (vs. si-FOXM1+UV group), ^##^*p* < 0.01, ^###^*p* < 0.001.

**Table 1:** Primers used in this study.

Primer name	Sequence (5′-3′)
SPAG5-F	TTGAGGCCCGTTTAGATACCA
SPAG5-R	GCTTTCCTTGGAGCAATGTAGTT
FOXM1-F	ATACGTGGATTGAGGACCACT
FOXM1-R	TCCAATGTCAAGTAGCGGTTG
IL-1*β*-F	ATGGCAGAAGTACCTAAGCTC
IL-1*β*-R	TTAGGAAGACACAAATTGCATGGTGAACTCAGT
IL-6-F	ATGAACTCCTTCTCCACAAGC
IL-6-R	CTACATTTGCCGAAGAGCCCTCAGGCTGGACTG
IL-18-F	GGCCTCTATTTGAAGATATGACTGATT
IL-18-R	CCTCTAGGCTGGCTATCTTTATACATAC
TNF*α*-F	AGGCGGTGCTTGTTCCTCA
TNF*α*-R	GTTCGAGAAGATGATCTGACTGCC
GAPDH-F	TGACTTCAACAGCGACACCCA
GAPDH-R	CACCCTGTTGCTGTAGCCAAA

## Data Availability

The data will be available on reasonable requests from the corresponding author.
